The article "The Clinical Efficacy and Risk Factors after Revision and Reconstruction of Anterior Cruciate Ligament" was retracted in 2023. Reasons: suspected computer-generated content; unreliable results or conclusions; lack of ethics approval or compliance; missing or withdrawn patient consent.

# The Clinical Efficacy and Risk Factors after Revision and Reconstruction of Anterior Cruciate Ligament

**DOI:** 10.1155/2021/6606492

**Published:** 2021-12-17

**Authors:** Shuai Miao, Shuoda Li, Zhonggao Wu, Hui Wang, Ming Li

**Affiliations:** ^1^Ningbo Haishu No. 2 Hospital Ningbo First Hospital Haishu Branch, Ningbo, Zhejiang, China; ^2^Ningbo Municipal Hospital of TCM, Ningbo, Zhejiang, China; ^3^Ningbo Beilun Changzheng Orthopaedic Hospital, Ningbo, Zhejiang, China

## Abstract

The aim of this study was to study the clinical efficacy and prognostic factors after revision and reconstruction of anterior cruciate ligament. All the patients who underwent the first revision of anterior cruciate ligament (ACL) reconstruction in the department of sports medicine from January 2001 to December 2015 were collected. The demographic information, the first revision and reconstruction information of ACL, and the information during the first ACL reconstruction were collected. A total of 335 cases were included. Lysholm score, Tegner activity score, and IKDC subjective score at the last follow-up were significantly higher than those before operation. Compared with graft failure caused by sports injury, the postoperative scores of patients with revision due to life accidents or initial reconstruction techniques were significantly lower (*P* < 0.05). The postoperative Lysholm score of patients with femoral canal drilling through the tibial canal was lower than that of patients with anterior internal approach. The postoperative IKDC score of patients who underwent medial meniscus suture at the same time was higher than that of patients without meniscus combined injury. ACL revision can improve the stability and function of knee joint. Compared with the revision caused by life accident or technical reasons of primary reconstruction surgery, the patients with graft failure caused by sports injury have better postoperative recovery. Medial meniscus suture and anterior internal approach drilling of the femoral bone canal have a statistically protective effect on the clinical function after ACL revision.

## 1. Introduction

Anterior cruciate ligament (ALC) reconstruction of the knee is one of the most extensive operations in the field of orthopaedic sports medicine. It can effectively improve the stability and function of the knee. However, the literature reports that 2% to 8% of patients fail after ACL reconstruction and may need ACL revision. In recent years, the number of ACL reconstruction operations is increasing, and the patients who need revision surgery are also increasing year by year [1, 2].

Previous studies have shown that the clinical effect after ACL revision is not as good as the initial reconstruction, and the graft failure rate and reoperation rate are also higher. Therefore, understanding the medium- and long-term clinical efficacy and its influencing factors after ACL revision surgery can optimize the treatment plan of revision surgery and scientifically adjust patients' expectations for postoperative efficacy, which is of great significance to improve knee function and patient satisfaction. Although there have been multicenter prospective registration studies in the world, there are few reports on the curative effect after ACL revision in Asia, and the number of clinical cases is small, and there is a lack of in-depth discussion on the influencing factors of curative effect [3, 4]. In this study, patients undergoing ACL revision were retrospectively followed up to evaluate the medium- and long-term clinical efficacy after revision, including graft failure rate, ipsilateral or contralateral knee reoperation rate, postoperative infection rate, and subjective score and, at the same time, the sex, age, BMI, duration of disease, causes of first failure, revision graft selection, and the effects of drilling method, combined injury, and treatment method of the femoral bone canal on the clinical curative effect [5].

## 2. Methods

### 2.1. Participants

The medical records of all patients who underwent ACL revision surgery in the Sports Medicine Department of the hospital from January 2001 to December 2015 were retrospectively studied. The inclusion criteria were as follows: (1) only ACL graft suture, partial bundle reconstruction, or original graft refixation were performed in the revision surgery; (2) primary reconstruction or revision reconstruction combined with posterior cruciate ligament (PCL) injury and lower limb fracture; (3) follow-up results <2 years; and (4) two or more revision operations. When analyzing the subjective scores of patients, the following exclusion criteria were added: (1) infection after primary reconstruction or revision reconstruction; (2) there were no follow-up results from the first revision to the second fracture of the graft, or the follow-up was less than 2 years.

### 2.2. Data Collection

The demographic information of patients and the first revision and reconstruction information of ACL (graft rupture time, failure reason, revision and reconstruction time, surgical technology, combined injury, and treatment method) were collected. The causes of failure are mainly divided into surgical technical errors, sports trauma, life accidents, traffic accidents, etc.; among them, surgical technical errors mainly include poor bone canal position, improper fixation or screw loosening, and improper graft selection; for specific classification methods, refer to the previous literature. For patients with initial ACL reconstruction in our department, the electronic medical record were reviewed and the information of initial ACL reconstruction is recorded in detail (initial fracture time, injury cause, injury mechanism, initial reconstruction time, surgical technique, combined injury, and treatment method); if it is carried out outside the hospital, as much initial reconstruction information as possible is collected by reviewing the inpatient records of the revision operation, and the patients were asked whether to keep the medical records of the initial reconstruction during the follow-up.

Patients who met the inclusion criteria were followed up, including pain visual analogue scale (VAS), Tegner activity level score, Lysholm score, knee subjective score of International Knee literature Committee, ipsilateral and contralateral knee injury, and hand operation after revision.

### 2.3. Statistical Analysis

All data were statistically analyzed using Stata software (22.0). Descriptive statistics are used to report patient demographic information, injury-related data, operation-related data, and clinical efficacy indicators. Categorical variables are expressed as quantity (%), continuous variables conforming to normal distribution are expressed as mean ± standard deviation, and continuous variables not conforming to normal distribution are expressed as median (minimum∼maximum). The *t* test or *χ*^2^ test for univariate analysis was used to explore the relationship between independent variables and clinical efficacy at the last follow-up. The independent variables with *P* < 0.20 in univariate analysis and the factors that may be related to functional score reported in the literature, such as gender, age, BMI, follow-up time, and preoperative baseline score, were included in multivariate analysis to determine the independent influencing factors of clinical efficacy. A paired *t* test was used to compare the subjective scores before and after operation. *P* < 0.05 was statistically significant. Due to the large time span of this study and the increased difficulty of follow-up, in order to test the representativeness of the research results, we also made a sensitivity analysis and compared the demographic information and revision surgery baseline information of lost patients and included patients.

## 3. Results

### 3.1. Patients

From January 2001 to December 2015, there were 335 cases of ACL first revision surgery meeting the research conditions. 166 cases were included in the actual follow-up, with a median follow-up time of 3.63 years. Among them, there were 128 males and 15 professional athletes. The average revision age was 28.56 years, and the average BMI was 26.41 kg/m^2^.

The most common reason for graft failure was the surgical technique, followed by sports injury and life accident.  Table 1 is the baseline characteristics of patients; 81 patients underwent initial reconstruction in our department. The common causes of revision were sports injury, followed by life accidents and surgical techniques. The most common sports in sports injuries are basketball and football. Autologous hamstring tendon and allograft were commonly used in the first ACL reconstruction, and autologous hamstring tendon and autologous bone patellar tendon bone were commonly used in the first ACL revision. A total of 32 patients were with surgery-related complication, and all the complications have been recovered as the follow-up.

### 3.2. Clinical Effect after First Revision of ACL

Infection occurred in 5 cases after revision, and the initial reconstruction was carried out in the external hospital. 41 patients underwent surgery again on the ipsilateral and contralateral knees during the follow-up period. Considering the impact of postoperative infection and secondary revision on clinical efficacy, this study only compared the preoperative and postoperative scores and analyzed the influencing factors of 160 patients who had no infection, no secondary revision, or not collected the follow-up results for more than 2 years before the secondary revision.  Table 2 is the comparison of clinical subjective scores before and after the first revision of ACL that showed that Lysholm score, Tegner activity level score, and IKDC subjective score at the last follow-up were significantly higher than those before operation (*P* < 0.05).

### 3.3. Influencing Factors of Clinical Efficacy after the First Revision of ACL

The influencing factors of Lysholm score after ACL revision include the reason of revision, the time from initial reconstruction to revision, and the drilling method of the femoral canal. Compared with the revision caused by sports injury, the postoperative Lysholm scores of patients with revision caused by life accident, traffic accident, or technical reasons decreased by 9.90 (95% CI: 1.49∼18.31), 18.67 (95% CI: 2.34∼35.00), and 8.53 (95% CI: 1.31∼15.75) (*P* < 0.05). For each additional year from initial reconstruction to revision, the postoperative Lysholm score decreased by 1.14 (95% CI: 0.03∼2.26) (*P*=0.045). The postoperative Lysholm score of patients with femoral canal drilling through the tibial canal was 11.18 lower than that of patients with an anterior internal approach (95% CI: 4.73∼17.63) (*P*=0.001). There was no significant difference in other factors.

The influencing factors of IKDC subjective score after ACL revision include the reason of revision and age at the time of revision. The older the revision age, the worse the postoperative score (*P*=0.042). Compared with the revision caused by sports injury, the postoperative IKDC subjective scores of patients with revision caused by life accident, traffic accident, or technical reasons were 10.35 (95% CI: 0.17∼20.54), 19.94 (95% CI: 2.94∼36.93), and 9.39 (95% CI: 1.03∼17.74) (*P* < 0.05). Medial meniscus suture had a protective effect (*P*=0.029). There was no significant difference in other factors.

The influencing factors of Tegner activity score after ACL revision include the reason of revision. Compared with the revision caused by sports injury, the postoperative Tegner activity score of patients with revision caused by life accident or technical reasons was 1.41 (95% CI: 0.10∼2.72) and 1.28 (95% CI: 0.14∼2.43) lower, respectively (*P* < 0.05).  Table 3 is the analysis of influencing factors of clinical efficacy after the first revision of ACL, and there was no significant difference in other factors in Table 3.

## 4. Discussion

ACL revision and reconstruction can improve knee function, and most patients can obtain satisfactory clinical curative effect. The literature shows that the excellent and good rate of ACL revision is 84%∼93%. The results of medium- and long-term follow-up after revision showed that Lysholm score, Tegner score, and IKDC subjective score were significantly higher than those before operation, and the stability of knee joint was significantly improved [6, 7].

However, the effect of revision surgery is generally less than that of primary reconstruction. The literature reported that the average IKDC score was 77 at 2 years after revision and 75 at 6 years after revision, which was 15∼20 points lower than that of the initial reconstruction [8]. In the 4.4-year follow-up results of this study, the average IKDC score was 80.23, which was close to the relevant domestic reports, but lower than the clinical efficacy of initial reconstruction reported in the literature. This may be because ACL rupture is often secondary to meniscus and/or cartilage injury. Many studies have found that the proportion of revision patients with meniscus injury or cartilage injury is as high as 36%∼75% and 24%∼67%, respectively. An international multicenter cohort study shows that 90% of ACL revision patients are complicated with at least one meniscus or grade 2 and above cartilage injury. In this study, the proportion is 93.61%, which is significantly higher than that of the initial reconstruction. Combined meniscus and cartilage injury will not only lead to pain and other symptoms and increase the risk of knee OA but also affect the stability of knee joint to some extent and seriously affect the function of knee joint [9].

In the medium- and long-term follow-up after revision, the graft failure rate was 2.7%∼33.3%, which was higher than 1.7%∼7.7% reported after the initial reconstruction. The median follow-up time was 3.63 years, the longest was 14.63 years, and the shortest was 2.03 years. During the follow-up period, the operation rate of ipsilateral and contralateral knee was 23.49%, of which the secondary revision rate was 3.01%, which was lower than 8.30% reported in China in the same period. Among the 5 patients who underwent secondary revision, the interval between 3 patients and the last revision was less than 1 year, and 2 of them were broken again due to playing basketball. Therefore, clinicians should strengthen the grasp of rehabilitation treatment and indications of return to movement after operation, so as to prevent graft rupture again and to avoid more serious degeneration of knee function [10].

Analyzing the clinical efficacy and prognostic factors of revision surgery can help clinicians and rehabilitation teachers better understand which patients have a poor prognosis, so as to further improve the scheme of surgical treatment and rehabilitation treatment, scientifically adjust the patients' expectations for the recovery of postoperative knee function, and achieve better objective treatment effect and clinical satisfaction [11]. Because the ACL revision rate is relatively low, it is difficult for a single center to collect large-sample cohort data. Although more ACL revision cases are included in this study, the time span is long, which is a certain challenge for carrying out prospective research. However, retrospective research will be difficult to determine the causal relationship between prognostic factors and curative effect due to selection, information, confounding, and other biases [12]. At present, many countries in the world have adopted multicenter or national system registration research. In the future, we hope to establish a domestic multicenter prospective cohort platform to collect rich and complete data as much as possible to further explore the factors affecting postoperative clinical efficacy and prognosis [13].

## 5. Conclusions

In conclusion, ACL revision and reconstruction can improve the stability of knee joint and significantly improve the function of knee joint. Compared with the revision caused by life accidents or technical reasons, the patients with revision caused by sports injury have better postoperative recovery. Suture of medial meniscus and drilling of the femoral canal through an anterior internal approach have statistically protective effects on clinical function after revision.

## Figures and Tables

**Table 1:** Patient baseline data.

Parameters	Included (*n* = 166)	Excluded (*n* = 169)	*P* value
Gender, *n* (%)			0.278
Male	128 (77.11)	99 (58.57)	
Female	38 (22.89)	41 (24.26)	
Professional athletes, *n* (%)	15 (9.04)	19 (11.24)	0.225
Age at revision/years	28.56 ± 7.60	27.04 ± 7.55	0.789
BMI/(kg/m^2^)	26.41 ± 3.73	24.31 ± 3.21	0.050
Interval between primary ACLR and revision/years, *M* (range)	2.78 (0.40–18.40)	3.17 (0.40–16.99)	0.841
Side, *n* (%)			0.897
Left knee	82 (49.40)	34 (20.11)	
Right knee	84 (50.60)	35 (20.71)	
Hospital of primary ACLR, *n* (%)			0.567
Index hospital	81 (48.80)	86 (50.88)	
Other hospitals	85 (51.20)	73 (43.19)	
Technique at primary ACLR, *n* (%)			0.184
Single bundle	70 (42.17)	85 (50.29)	
Double bundle	10 (6.02)	8 (4.73)	
Unknown	86 (51.81)	73 (43.19)	

**Table 2:** Comparison of clinical subjective scores before and after the first revision of ACL.

Patient-reported outcomes	Preoperation	Last follow-up	*P* value
Tegner	4.39 ± 1.78	4.87 ± 1.75	<0.001
IKDC	68.78 ± 15.01	81.23 ± 13.30	<0.001
Lysholm	78.51 ± 21.22	89.64 ± 14.35	<0.001

**Table 3:** Analysis of influencing factors of clinical efficacy after the first revision of ACL.

Predictors	Lysholm		IKDC subjective score		Tegner	
	95%CI	*P* value	95%CI	*P* value	95%CI	*P* value
*Gender*						
Male	Reference		Reference		Reference	
Female	−0.98 (−8.72, 6.75)	0.801	−3.97 (−13.08, 5.15)	0.384	−0.08 (−1.62, 1.46)	0.917
Age at revision	−0.35 (−0.95, 0.25)	0.248	−0.91 (−1.78, −0.03)	0.042	−0.04 (−0.15, 0.07)	0.426
BMI	−0.25 (−1.09, 0.61)	0.571			0.07 (−0.07, 0.21)	0.35

*Cause of graft failure*						
Sports	Reference		Reference		Reference	
Daily activities	−9.90 (−18.31, −1.49)	0.022	−10.35 (−20.54, −0.17)	0.047	−1.41 (−2.72, −0.10)	0.035
Traffic accident	−18.67 (−35.00, −2.34)	0.026	−19.94 (−36.93, −2.94)	0.023	−2.45 (−5.12, 0.22)	0.071
Technical	−8.53 (−15.75, −1.31)	0.021	−9.39 (−17.74, −1.03)	0.029	−1.28 (−2.43, −0.14)	0.031

## Data Availability

The simulation experiment data used to support the findings of this study are available from the corresponding author upon request.
